# Exosome Derived from Human Neural Stem Cells Improves Motor Activity and Neurogenesis in a Traumatic Brain Injury Model

**DOI:** 10.1155/2022/6409346

**Published:** 2022-08-12

**Authors:** Mahsa Abedi, Mehrdad Hajinejad, Fereshteh Atabi, Sajad Sahab-Negah

**Affiliations:** ^1^Department of Biochemistry and Biophysics, Faculty of Advanced Sciences and Technology, Tehran Medical Sciences, Islamic Azad University, Tehran, Iran; ^2^Shefa Neuroscience Research Center, Khatam Alanbia Hospital, Tehran, Iran; ^3^Department of Anatomy and Cell Biology, School of Medicine, Mashhad University of Medical Sciences, Mashhad, Iran; ^4^Student Research Committee, Mashhad University of Medical Sciences, Mashhad, Iran; ^5^Neuroscience Research Center, Mashhad University of Medical Sciences, Mashhad, Iran; ^6^Department of Neuroscience, Faculty of Medicine, Mashhad University of Medical Sciences, Mashhad, Iran

## Abstract

Traumatic brain injury (TBI) is a leading cause of mortality and long-lasting disability globally. Although novel treatment options have been investigated, no effective therapeutic opportunities for TBI exist. Accumulating studies demonstrated that the paracrine mechanisms of stem cells may allow them to orchestrate regenerative processes after TBI. So far, very little attention has been paid to the beneficial effects of human neural stem cells (hNSCs) in comparison to their exosomes as a paracrine mechanism. This study is aimed at comparing the effect of hNSCs with their exosomes in a TBI model. For in vitro assessments, we cultured hNSCs using the neurosphere method and isolated hNSC-derived exosomes from culture supernatants. For in vivo experiments, male rats were divided into three groups (*n* = 8/group): TBI group: rats were subjected to a unilateral mild cortical impact; hNSC group: rats received a single intralesional injection of 2 × 10^6^ hNSCs after TBI; and exosome group: rats received a single intralesional injection of 63 *μ*g protein of hNSC-derived exosomes after TBI. Neurological assessments, neuroinflammation, and neurogenesis were performed at the predetermined time points after TBI. Our results indicated that the administration of exosomes improved the neurobehavioral performance measured by the modified neurological severity score (mNSS) on day 28 after TBI. Furthermore, exosomes inhibited the expression of reactive astrocytes as a key regulator of neuroinflammation marked by GFAP at the protein level, while enhancing the expression of Doublecortin (DCX) as a neurogenesis marker at the mRNA level. On the other hand, we observed that the expression of stemness markers (SOX2 and Nestin) was elevated in the hNSC group compared to the exosome and TBI groups. To sum up, our results demonstrated that the superior effects of exosomes versus parent hNSCs could be mediated by improving mNSS score and increasing DCX in TBI. Considerably, more work will need to be done to determine the beneficial effects of exosomes versus parent cells in the context of TBI.

## 1. Introduction

Traumatic brain injury (TBI) is caused by a mechanical force on the brain tissue [1]. TBI severity can be classified into severe, moderate, and mild by scores on the Glasgow Coma Scale that can cause substantial neurological disabilities and mental distress [2]. TBI has been estimated to create an alarming rate in the United States with 10 million cases annually and become the third leading cause of death worldwide [3]. TBI does not have a single pathophysiological appearance; it is a multimodal complex disease process in which primary and secondary injuries induce numerous pathological changes to the brain parenchyma [1, 2]. Proinflammatory cytokines secreted by glial cells (i.e., astrocytes and microglia) play important roles in the pathogenesis of TBI [4]. Glutamate toxicity and oxidative stress are other prominent molecular mechanisms that induce cell death and increase the severity of TBI [1, 5]. Despite global efforts to find out effective treatment, there is no cure treatment for TBI [6]. During the last decades, stem cell treatment strategies have shown promising results in experimental and some clinical studies [7]. In recent years, different types of stem cells, such as mesenchymal stem cells (MSCs), hematopoietic stem cells, umbilical cord stem cells, and neural stem cells (NSCs), have been investigated in the course of TBI [6]. For example, transplantation of NSCs promoted functional recovery after a TBI model by increasing synaptic density [8]. Recently, our team showed that NSC therapy in conjunction with nanocurcumin increased recovery from TBI by decreasing astrogliosis and its downstream neuroinflammatory pathways [9]. However, several challenges remain to be overcome before stem cell therapy can become a reality for patients [10, 11]. For example, immune responses after transplantation, oncogenic properties, low neuronal differentiation capacity, and low cell engraftment should be carefully assessed [12]. Recently, bystander effects of stem cells (i.e., paracrine mechanisms) have been introduced as an alternative approach to stem cell therapy [13, 14]. Among different bystander mechanisms, a new mechanism for intercellular communication has emerged which involves the intercellular transfer of exosomes [15]. Up to now, numerous studies have been done on the beneficial effects of exosomes derived from MSCs in neurological disorders. They presented reasonable explanations of why exosomes are valuable therapeutic agents for TBI [16, 17]. Exosomes are nanosized extracellular vesicles (30-100 nm) that carry cell-specific cargos of proteins, lipids, and RNA (mRNA, noncoding RNA, etc.) [18]. Exosomes can affect the physiological function of target cells by regulating gene expression or protein synthesis [17]. It should be noted that there has been little discussion about the beneficial effects of exosomes derived from human neural stem cells (hNSCs) in the course of TBI. Hence, we hypothesized that exosomes derived from hNSCs could be advantageous for TBI and thus offer a better way for treatments. Therefore, the present study primarily investigated whether hNSC-derived exosomes could improve functional recovery and pathological changes after TBI. More essentially, we compared the beneficial effects of hNSC-derived exosomes with hNSCs in an experimental brain injury model for the first time.

## 2. Materials and Methods

### 2.1. In Vitro Assessments

#### 2.1.1. Culture of hNSCs

hNSCs were purchased from the Biobank of Neuroscience Department of Mashhad University of Medical Sciences. hNSCs were cultured in Dulbecco's Modified Eagle Medium/Nutrient Mixture F-12 (DMEM/F-12) (Gibco, Germany) containing 1.5% fetal bovine serum (FBS) (Gibco, Germany), 0.5% penicillin-streptomycin (Pen/Strep) (Gibco, Germany), 0.5% L-glutamine (Gibco, Germany), 0.5% B27 (Gibco, Germany), 0.25% N2 (Gibco, Germany), and 20 ng/mL epidermal growth factor (EGF) (Sigma, Germany).

The hNSCs were characterized with ICC staining against nestin and SOX2 proteins as a neural stem cell marker.

### 2.2. Isolation and Characterization of Exosomes

#### 2.2.1. Isolation of Exosome

To isolate exosomes from hNSCs, the hNSCs were cultured in a serum-free media for 48 h, and then, the supernatant was collected. Next, debris and apoptotic parts of cells were removed by centrifugation. After that, the supernatant was incubated overnight at 4°C with Exosomes Isolation Kit (Invitrogen, 4478359), according to the manufacturer protocol, which was followed by centrifugation at 10000 g for 1 h. Finally, the supernatant was discarded, and the pellets were suspended in 100–1000 *μ*L of PBS and stored in a −80°C refrigerator. The exosome concentration was determined with a BCA Protein Assay Kit (Parstous, A101251).

### 2.3. Size Characterization of Exosomes

#### 2.3.1. Transmission Electron Microscope (TEM)

The double-layer membrane structure exosomes were detected by TEM. For this, the exosome pellet was dissolved in deionized water (DW). Then, negative staining was performed using 10 *μ*L of exosome suspension solution that was loaded on the grid and stained with 2% uranyl acetate. Finally, the samples were dried and directly put on the electron microscopy grid and visualized by a TEM microscopy (Zeiss Leo 912).

#### 2.3.2. Scanning Electron Microscope (SEM)

The morphology of exosomes was characterized by SEM. The exosome pellet was suspended in DW and fixed in a 2% paraformaldehyde aqueous solution. Next, 5 *μ*L of exosomes solution was loaded on an aluminum foil and coated with 2-5 nm of gold by sputtering (20 mA for 150 s). Finally, SEM was performed under low beam energies (5.0-10.0 kV) (TSCAN MIRA3).

#### 2.3.3. Dynamic Light Scattering (DLS)

DLS is a well-established technique for measuring the size and size distribution of molecules and particles [19]. For analysis of the size of exosomes, purified isolated exosomes were dissolved in DW and immediately analyzed with Cordouan (Vasco3, France).

### 2.4. In Vivo Assessments

#### 2.4.1. Animal Ethical Statement

Male Wistar rats (220–250 g) were purchased from the Animal Laboratory of Medical School of Mashhad University of Medical Sciences. All experiment procedures were performed according to the National Institutes of Health Guidelines and were approved by the Animal Use and Ethics Committee of Mashhad University of Medical Sciences Animals were kept with free access to water and food, temperature of 23 ± 2°C, relative humidity of 65 ± 10%, and 12 h light/dark cycle.

#### 2.4.2. Animal Model of Moderate Traumatic Brain Injury (mTBI)

After intraperitoneal administration of ketamine (20 mg/kg) and xylazine (10 mg/kg), rats were fixed in a stereotaxic frame. The scalp was opened by a drill. The dura mater was removed (A‐P = 0 mm, M‐L = 1.5 mm, and DV: 2 mm), and a cavity was created by inserting a rotary biopsy punch (2 mm diameter; Miltex, USA). Rats were housed in separate cages after surgery and kept in standard condition.

#### 2.4.3. Animal Group and Administration of hNSCs and Exosomes

After TBI, male rats were randomly divided into three groups (*n* = 8/group): TBI group: rats were subjected to a unilateral mild cortical impact; hNSC group: rats received a single intralesional injection of 2 × 10^6^ hNSCs after TBI; and exosome group: rats received a single intralesional injection of 63 *μ*g protein of exosomes after TBI.

#### 2.4.4. Behavioral Assessments

The neurological function was evaluated using the modified neurological severity score (mNSS) test at predetermined time points (i.e., 7, 14, 21, and 28 days) after TBI. To include animals with moderate severity, the mNSS test was also used on day 1 for confirming. The open-field test was performed to measure general locomotor activity levels on days 8 and 28 after TBI. Rotarod test was also used to evaluate the motor coordination on days 5 and 10 after TBI.

#### 2.4.5. qRT-PCR Analysis

To analyze the inflammatory and neurogenic gene in response to exosome and stem cell therapy, a reverse transcription-polymerase chain reaction (qRT-PCR) was performed. The total RNA was extracted from brain cortex by a total RNA extraction kit (Pars-151001). A total of 1 *μ*g of RNA was reverse transcribed into cDNA using the easy cDNA reverse transcription kit (Pars tous-5301142). Next, qRT-PCR real-time was performed by PCR thermal cycler (LightCycler System; Roche Diagnostics Corp., Indianapolis, IN, USA) using qPCR SYBR Green master mix (Amplicon-A323402-25). *β*-Actin was used as an internal control to normalize the data. The primers used in our study are listed in Table 1.

#### 2.4.6. Immunohistochemistry

To evaluate astrogliosis, differences in GFAP labeling in reactive astrocytes damaged by TBI were assessed by the immunohistochemistry method. The astrocytes marked with GFAP were detected by immunohistochemistry. Rats were anesthetized with an intraperitoneal administration of ketamine (20 mg/kg) and xylazine (10 mg/kg) on day 28 after injury. The brain samples were fixed in 10% formaldehyde. The brain tissue was embedded in paraffin and cut into 5 *μ*m thick sections. Next, the sections were stained for GFAP by using a preembedding immunohistochemistry procedure.

After deparaffinization, antigen retrieval was performed in PBS at 100°C temperature and followed by endogenous peroxidase using 3% H_2_O_2_. Then, all brain sections were blocked with 5% normal goat serum for 30 min and incubated with a specific primary antibody, rabbit anti-GFAP (1 : 2000; ab7260, Abcam, USA), at 4°C overnight. On the following day, brain sections were incubated with horseradish peroxidase- (HRP-) conjugated goat anti-rabbit (1 : 1000; ab6721, Abcam, USA) as the secondary antibody at room temperature for 1 h. Next, sections were counterstained with hematoxylin and mounted on glass slides. Finally, the sections were evaluated with a bright field microscope (Olympus 30 × 23, Japan).

#### 2.4.7. Data Analysis

All data were expressed as means ± SEM. All data were analyzed with IBM SPSS Statistics v22.0. For comparison of behavioral data between groups, two-way ANOVA analyses were performed followed by post hoc analyses using the Bonferroni procedure for multiple comparisons. One-way ANOVA, followed by the Tukey post hoc test, was used to assess the significant differences among different groups for other experiments. A *P* value less than 0.05 was considered statistically significant.

## 3. Results

### 3.1. Characterization of hNSCs

The stemness properties of human NSCs were detected by neurosphere formation and nestin-positive cells. Our results showed that isolated hNSCs had great potential for self-renewal by forming a neurosphere (Figure 1(a)). We also observed that the majority of stem cells expressed nestin as a stem cell marker (Figure 1(b)).

### 3.2. Characterization of Exosomes

To identify the size of exosomes, SEM and TEM techniques were used. Data from SEM imaging showed that hNSC-derived exosomes were spherical nanoparticles (Figure 2(a)). Furthermore, the size range of exosomes was detected between 20 and 100 nanometres by TEM (Figure 2(b)). In addition, the size and size distribution of exosome were assessed by DLS. Our results indicated that the mean size and polydispersity index of exosomes isolated from human NSCs were 101.49 nm and 0.43, respectively (Figure 2(c)).

### 3.3. Behavioral Assessments

Neurological deficits were measured by mNSS score. According to our results, administration of hNSCs and exosomes significantly reduced the mNSS score compared to the TBI group at 7, 14, 21, and 28 days after injury (Figure 3(a)). Moreover, neurological impairments were remarkably reduced in the exosome group compared to the hNSC group on day 28 after injury (Figure 3(a)). However, there was no significant difference in travel of distance measured by OF (Figure 3(b)) and latency to fall off estimated by rotarod test (Figure 3(c)) between groups.

### 3.4. Exosomes vs. Their Parental Stem Cells on Stemness and Neurogenesis Markers

To evaluate and compare the effects of exosomes vs. their parental stem cells on regeneration processes after TBI, the mRNA expression levels of SOX2, Nestin, and Doublecortin (DCX) were evaluated.

Our results indicated that the expression of SOX2 and Nestin was significantly increased in the hNSC group compared to the TBI group (Figures 4(a) and 4(b)). We also observed that the mRNA expression of Nestin was significantly increased in the hNSC group compared to the exosome group (Figure 4(b); *P* < 0.001). On the other hand, the mRNA expression level of DCX as a neurogenesis marker was significantly enhanced in the exosome group compared to the TBI group (Figure 4(c); *P* < 0.05).

### 3.5. HNSCs vs. Their Exosomes on Astrogliosis after TBI

GFAP is expressed in astrocytes that substantially increased in response to TBI [20, 21]. The protein level of GFAP in the perilesional site was significantly reduced in the hNSC and exosome groups compared to the TBI group (Figure 5; *P* < 0.05).

## 4. Discussion

In the current study, we showed that the administration of hNSC-derived exosomes improved neurobehavioral performance after TBI. Furthermore, exosomes decreased the expression of reactive astrocytes marked by GFAP as a key regulator of neuroinflammation at the protein level, while increasing the mRNA expression level of DCX as a neurogenesis marker. However, the mRNA expression of SOX2 and Nestin as the stemness markers was elevated in the hNSC group compared to the exosome and TBI groups. The empirical findings in this study provide a new understanding of the beneficial effects of exosomes compared to their parent cells as a cell-free treatment strategy in the course of TBI. TBI has complex pathological changes that include primary and secondary injuries [22]. A variety of cellular and molecular events, such as neuronal loss, accumulation of intracellular, mitochondrial dysfunction, oxidative stress, neuroinflammation, and necrotic debris, take place after TBI [23, 24]. Due to the complex cascades of events, there is no effective therapeutic strategy for TBI [25]. Thus, finding a novel therapeutic strategy for promoting pathological changes is warranted.

Stem cell-derived exosomes improve functional neurologic recovery and diminish spatial learning impairments after TBI [17, 20]. Potential mechanisms for exosome therapy as a cell-free-based therapeutic option can be taken place by improving angiogenesis and neurogenesis and suppressing neuroinflammation [26]. Because the vast majority of studies have focused on the potential effects of MSC-derived exosomes, still little is known about the effects of exosomes derived from other cell sources in the course of TBI [27, 28]. For example, there is little study on exosomes derived from human neural stem cells in the course of TBI [29]; therefore, having adequate data on the effects of exosomes compared to their parent NSCs gives us new insights to understand the underlying mechanisms of paracrine effects of hNSCs. In the current study, we compared the beneficial effects of exosomes with their parent hNSCs on functional recovery, astrogliosis, and neurogenesis after the TBI model. By the present results, previous studies have demonstrated that exosomes derived from stem cells improved functional recovery after TBI [17, 22]. Consistent with the literature [23, 24], this research found that exosomes increased neurogenesis markers after TBI.

Another important finding of our study was that astrogliosis marked by GFAP at the protein level was significantly decreased in the exosome group. We now know from lots of studies that increased reactive astrocytes play a crucial role in the pathogenesis of TBI patients and preclinical animal models [30]. Decreasing astrogliosis by exosomes seems to be consistent with other research which found that exosomes derived from MSCs could attenuate neuroinflammation through glial suppression [31, 32]. Our findings suggest further research on neuroinflammatory pathways and their downstream signals in response to exosomes after TBI. However, the major limitation of the current study was the low concentration of exosomes which may constitute the object of future studies. Another limitation was that we assessed the DCX as a neurogenesis marker at the mRNA level; therefore, further research is suggested to evaluate this marker at the protein level for having a strong conclusion.

## 5. Conclusion

Taken together, our study provides evidence to support the ability of hNSC-derived exosomes as a novel approach in cell-free therapy and become an important therapeutic tool after brain injury. Our results indicated that hNSC-derived exosomes have superior effects vs. parental cells in terms of sensorimotor functional recovery and neurogenesis after TBI. As a result, to develop a full picture of the beneficial effects of the hNSC-derived exosome, further studies will need to be undertaken.

## Figures and Tables

**Figure 1:** Culture and characterization of hNSCs. (a) Phase-contrast images of neurosphere formation from single hNSCs. (b) Immunocytochemistry staining for Nestin (green) in NSC culture.

**Figure 2:** Characterization of the hNSC-derived exosomes. (a) Scanning electron microscopy image of exosomes. Scale bar: 200 nm. (b) Transmission electron microscopy image of exosomes that show nanoscale of exosomes. Scale bar: 100 nm. (c) The size and size distribution of purified exosomes which derived from hNSCs were measured by nanoparticle tracking analysis. The mean number and polydispersity index hNSC-derived exosomes were 101.49 nm and 0.43, respectively.

**Figure 3:** Effect of hNSCs and their exosomes on behavioral assessments. The sensorimotor and functional recovery were evaluated by mNSS (a), open field (b), and rotarod test (c). hNSCs and exosomes significantly reduced the mNSS score. There was no observed difference in the open field and rotarod tests between groups. Data are shown as the mean ± SEM (*n* = 10/group).

**Figure 4:** RT-PCR was used to evaluate the mRNA levels of SOX2 (a), Nestin (b), and DCX (c). Transplantation of hNSCs increased greatly the levels of SOX2 and Nestin after injury. The administration of the exosome increased the mRNA level of DCX. Data are shown as the mean ± SEM (*n* = 5/group).

**Figure 5:** The protein expression of GFAP was evaluated after injury by IHC to detect reactive astrocytes. The hNSCs and exosome markedly reduced the activation of astrocytes after TBI. Data are shown as the mean ± SEM (*n* = 5/group).

**Table 1:** Primer list.

Gene name	Primer	
	Forward	Reverse
*β*-Actin	GCGCAAGTACTCTGTGTGG	CATCGTACTCCTGCTTGCTG
Nestin	CTGAGGCCTCTCTTCTTCCA	ACTCCTGTACCGGGTCTCCT
SOX2	CCCACCTACAGCATGTCCTA	TGGAGTGGGAGGAAGAGGTA
DCX	GCTGACCTGACTCGATCCTT	CCGACCAGTTGGGATTGACAT

## Data Availability

There is no data availability.

## References

[1] Ladak A. A., Enam S. A., Ibrahim M. T. (2019). A review of the molecular mechanisms of traumatic brain injury. *World Neurosurgery*.

[2] Pavlovic D., Pekic S., Stojanovic M., Popovic V. (2019). Traumatic brain injury: neuropathological, neurocognitive and neurobehavioral sequelae. *Pituitary*.

[3] Hyder A. A., Wunderlich C. A., Puvanachandra P., Gururaj G., Kobusingye O. C. (2007). The impact of traumatic brain injuries: a global perspective. *NeuroRehabilitation*.

[4] Alam A., Thelin E. P., Tajsic T. (2020). Cellular infiltration in traumatic brain injury. *Journal of Neuroinflammation*.

[5] Kappy N. S., Chang S., Harris W. M. (2018). Human adipose-derived stem cell treatment modulates cellular protection in both in vitro and in vivo traumatic brain injury models. *Journal of Trauma and Acute Care Surgery*.

[6] Zhou Y., Shao A., Xu W., Wu H., Deng Y. (2019). Advance of stem cell treatment for traumatic brain injury. *Frontiers in Cellular Neuroscience*.

[7] Weston N. M., Sun D. (2018). The potential of stem cells in treatment of traumatic brain injury. *Current Neurology and Neuroscience Reports*.

[8] Xiong L.-L., Hu Y., Zhang P. (2018). Neural stem cell transplantation promotes functional recovery from traumatic brain injury via brain derived neurotrophic factor-mediated neuroplasticity. *Molecular Neurobiology*.

[9] Narouiepour A., Ebrahimzadeh-bideskan A., Rajabzadeh G., Gorji A., Negah S. S. (2022). Neural stem cell therapy in conjunction with curcumin loaded in niosomal nanoparticles enhanced recovery from traumatic brain injury. *Scientific Reports*.

[10] Zakrzewski W., Dobrzyński M., Szymonowicz M., Rybak Z. (2019). Stem cells: past, present, and future. *Stem Cell Research & Therapy*.

[11] Yamanaka S. (2020). Pluripotent stem cell-based cell therapy--promise and challenges. *Cell Stem Cell*.

[12] Sun M. K., Passaro A. P., Latchoumane C. F. (2020). Extracellular vesicles mediate neuroprotection and functional recovery after traumatic brain injury. *Journal of Neurotrauma*.

[13] Widera D. (2021). Recent advances in translational adipose-derived stem cell biology. *Biomolecules*.

[14] Hajinejad M., Sahab-Negah S. (2021). Neuroinflammation: the next target of exosomal microRNAs derived from mesenchymal stem cells in the context of neurological disorders. *Journal of Cellular Physiology*.

[15] Van Niel G., Porto-Carreiro I., Simoes S., Raposo G. (2006). Exosomes: a common pathway for a specialized function. *Journal of Biochemistry*.

[16] Zhang Y., Zhang Y., Chopp M., Zhang Z. G., Mahmood A., Xiong Y. (2020). Mesenchymal stem cell–derived exosomes improve functional recovery in rats after traumatic brain injury: a dose-response and therapeutic window study. *Neurorehabilitation and Neural Repair*.

[17] Zhong D., Cao Y., Li C. J. (2020). Neural stem cell-derived exosomes facilitate spinal cord functional recovery after injury by promoting angiogenesis. *Experimental Biology and Medicine*.

[18] Chen J., Chopp M. (2018). Exosome therapy for stroke. *Stroke*.

[19] Zhang W., Peng P., Kuang Y. (2016). Characterization of exosomes derived from ovarian cancer cells and normal ovarian epithelial cells by nanoparticle tracking analysis. *Tumor Biology*.

[20] Zwirner J., Lier J., Franke H. (2021). GFAP positivity in neurons following traumatic brain injuries. *International Journal of Legal Medicine*.

[21] Yue J. K., Yuh E. L., Korley F. K. (2019). Association between plasma GFAP concentrations and MRI abnormalities in patients with CT-negative traumatic brain injury in the TRACK-TBI cohort: a prospective multicentre study. *The Lancet Neurology*.

[22] Thapa K., Khan H., Singh T. G., Kaur A. (2021). Traumatic brain injury: mechanistic insight on pathophysiology and potential therapeutic targets. *Journal of Molecular Neuroscience*.

[23] Crupi R., Cordaro M., Cuzzocrea S., Impellizzeri D. (2020). Management of traumatic brain injury: from present to future. *Antioxidants*.

[24] Sulhan S., Lyon K. A., Shapiro L. A., Huang J. H. (2020). Neuroinflammation and blood–brain barrier disruption following traumatic brain injury: pathophysiology and potential therapeutic targets. *Journal of Neuroscience Research*.

[25] Dekmak A., Mantash S., Shaito A. (2018). Stem cells and combination therapy for the treatment of traumatic brain injury. *Behavioural Brain Research*.

[26] Yang Y., Ye Y., Su X., He J., Bai W., He X. (2017). MSCs-derived exosomes and neuroinflammation, neurogenesis and therapy of traumatic brain injury. *Frontiers in Cellular Neuroscience*.

[27] Reza-Zaldivar E. E., Hernández-Sapiéns M. A., Minjarez B., Gutiérrez-Mercado Y. K., Márquez-Aguirre A. L., Canales-Aguirre A. A. (2018). Potential effects of MSC-derived exosomes in neuroplasticity in Alzheimer’s disease. *Frontiers in Cellular Neuroscience*.

[28] Gorabi A. M., Kiaie N., Barreto G. E., Read M. I., Tafti H. A., Sahebkar A. (2019). The therapeutic potential of mesenchymal stem cell–derived exosomes in treatment of neurodegenerative diseases. *Molecular Neurobiology*.

[29] Luo H., Ye G., Liu Y. (2022). miR-150-3p enhances neuroprotective effects of neural stem cell exosomes after hypoxic-ischemic brain injury by targeting CASP2. *Neuroscience Letters*.

[30] Michinaga S., Koyama Y. (2021). Pathophysiological responses and roles of astrocytes in traumatic brain injury. *International Journal of Molecular Sciences*.

[31] Zhang Y., Chopp M., Meng Y. (2015). Effect of exosomes derived from multipluripotent mesenchymal stromal cells on functional recovery and neurovascular plasticity in rats after traumatic brain injury. *Journal of Neurosurgery*.

[32] Zhang Y., Chopp M., Zhang Z. G. (2017). Systemic administration of cell-free exosomes generated by human bone marrow derived mesenchymal stem cells cultured under 2D and 3D conditions improves functional recovery in rats after traumatic brain injury. *Neurochemistry International*.

